# CCR2 Gene Deletion and Pharmacologic Blockade Ameliorate a Severe Murine Experimental Autoimmune Neuritis Model of Guillain-Barré Syndrome

**DOI:** 10.1371/journal.pone.0090463

**Published:** 2014-03-14

**Authors:** Furong Yuan, Nejla Yosef, Chetan Lakshmana Reddy, Ailing Huang, Sharon C. Chiang, Hafiza Rahman Tithi, Eroboghene E. Ubogu

**Affiliations:** 1 Neuromuscular Immunopathology Research Laboratory, Department of Neurology, Baylor College of Medicine, Houston, Texas, United States of America; 2 Department of Molecular Physiology and Biophysics, Baylor College of Medicine, Houston, Texas, United States of America; 3 Department of Statistics, Rice University, Houston, Texas, United States of America; University of Edinburgh, United Kingdom

## Abstract

The molecular determinants and signaling pathways responsible for hematogenous leukocyte trafficking during peripheral neuroinflammation are incompletely elucidated. Chemokine ligand/receptor pair CCL2/CCR2 has been pathogenically implicated in the acute inflammatory demyelinating polyradiculoneuropathy variant of Guillain-Barré syndrome (GBS). We evaluated the role of CCR2 in peripheral neuroinflammation utilizing a severe murine experimental autoimmune neuritis (sm-EAN) model. Sm-EAN was induced in 8–12 week old female SJL CCR2 knockout (CCR2KO), heterozygote (CCR2HT) and wild type (CCR2WT) mice, and daily neuromuscular severity scores and weights recorded. *In vitro* and *in vivo* splenocyte proliferation and cytokine expression assays, and sciatic nerve Toll-like receptor (TLR) 2, TLR4 and CCL2 expression assays were performed to evaluate systemic and local innate immune activation at disease onset. Motor nerve electrophysiology and sciatic nerve histology were also performed to characterize the inflammatory neuropathy at expected peak severity. To further determine the functional relevance of CCR2 in sm-EAN, 20 mg/kg CCR2 antagonist, RS 102895 was administered daily for 5 days to a cohort of CCR2WT mice following sm-EAN disease onset, with efficacy compared to 400 mg/kg human intravenous immunoglobulin (IVIg). CCR2KO mice were relatively resistant to sm-EAN compared to CCR2WT and CCR2HT mice, associated with attenuated peripheral nerve demyelinating neuritis. Partial CCR2 gene deletion did not confer any protection against sm-EAN. CCR2KO mice demonstrated similar splenocyte activation or proliferation profiles, as well as TLR2, TLR4 and CCL2 expression to CCR2WT or CCR2HT mice, implying a direct role for CCR2 in sm-EAN pathogenesis. CCR2 signaling blockade resulted in rapid, near complete recovery from sm-EAN following disease onset. RS 102895 was significantly more efficacious than IVIg. CCR2 mediates pathogenic hematogenous monocyte trafficking into peripheral nerves, with consequential demyelination in sm-EAN. CCR2 is amenable to pharmacologic blockade, making it a plausible drug target for GBS.

## Introduction

The acute inflammatory demyelinating polyradiculoneuropathy (AIDP) variant of Guillain-Barré syndrome (GBS) is the most common immune-mediated peripheral neuritis in developed countries. AIDP remains a major cause of morbidity and mortality despite current treatments. AIDP is pathologically characterized by macrophage-induced demyelination associated with intense T-cell and B-cell infiltration into peripheral nerves and nerve roots [1], [2]. The molecular determinants or signaling mechanisms relevant to pathogenic leukocyte trafficking into peripheral nerves during immune-mediated demyelination are not fully known. Several observational studies have implicated chemokines and other cytokines in GBS pathogenesis [3], [4]. Chemokines and their G-protein coupled receptors (GPCRs) are of particular interest, as they facilitate chemotaxis across concentration gradients *in vitro* and haptotaxis during inflammation *in vivo*.

Furthermore, as GPCRs, chemokine receptors are amenable to pharmacologic modulation as seen with plexirafor (a CXCR4 antagonist that functions as a hematopoietic stem cell mobilizer, used in combination with granulocyte-colony stimulating factor to mobilize hematopoietic stem cells to the peripheral blood for collection and subsequent autologous transplantation in patients with non-Hodgkin's lymphoma and multiple myeloma) and maraviroc (a selective, slowly reversible small molecular CCR5 antagonist that prevents CCR5-tropic human immunodeficiency virus [HIV]-1 entry into human cells by blocking the interaction between CCR5 and HIV-1 gp120). Although the literature on the chemokine biology of GBS is relatively sparse, several studies suggest potential roles for CCL2/CCR2, CCL5/CCR5 and CXCL10/CXCR3 signaling in AIDP pathogenesis [3].

Of particular interest is a study that focused on serum and peripheral nerve biopsy CCL2 and CCR2 expression in 38 GBS patients compared to 17 healthy controls. This study demonstrated peak serum CCL2 levels at maximum GBS disease severity, with the highest levels observed in the most disabled patients. CCL2 was also observed on epineurial and endoneurial vessels, infiltrating leukocytes, Schwann cells and the endoneurial extracellular matrix. Fewer circulating CCR2+ mononuclear cells were seen in GBS patients compared to controls, with CCR2+ cells detected in GBS patient peripheral nerve biopsies. The data implied that CCL2 may facilitate pathogenic CCR2+ mononuclear leukocyte infiltration into peripheral nerves in GBS [5]. However, the relationship between circulating blood and endoneurial CCL2 levels is unknown. It is provocative to speculate that inflammatory changes at the blood-nerve barrier may be associated with increased nerve root cerebrospinal fluid (CSF) chemokine secretion, based on observational data that showed a correlation between CSF CXCL10 and CCL2 levels and increased CSF: plasma albumin ratios in GBS [6]. It is also plausible that CCL2 secreted within inflamed peripheral nerves is released directly into the bloodstream via blood-nerve barrier efflux mechanisms. Nonetheless, the former referenced study supports the notion that CCL2/CCR2 dependent signaling may be associated with GBS pathogenesis, providing rationale for mechanistic evaluation.

Functional studies relevant to human AIDP can be studied using a representative animal model, experimental autoimmune neuritis (EAN) prior to clinical trials [7]. A recently characterized mouse model, severe murine EAN (sm-EAN) is a reliably robust AIDP animal model due to its high induction rates, as well as demonstrated electrophysiologic and pathologic correlation with disease severity. 8-12-week-old female SJL mice are immunized with bovine peripheral nerve myelin (BPNM) emulsified in complete Freund Adjuvant (CFA), using pertussis toxin and recombinant mouse interleukin-12 as a co-adjuvants, inducing a severe monophasic primarily demyelinating polyneuritis with some associated axonal loss [8]–[10]. Since hematogenous monocytes/macrophages are predominantly CCR2+ [11] and are the most prevalent leukocyte subpopulation observed in peripheral nerves in AIDP and murine EAN models [9], [12], [13], we sought to deduce whether CCR2 is directly relevant to sm-EAN pathogenesis using gene knockout and pharmacologic blockade strategies. This work has translational potential as knowledge obtained from this study could guide the process of developing target-specific anti-inflammatory therapies for peripheral neuroinflammation.

## Materials and Methods

The work described was ethically carried out based on the Uniform Requirements for manuscripts submitted to Biomedical journals.

### Experimental mice and polymerase chain reaction genotyping

All animal procedures were reviewed and approved by the Baylor College of Medicine (BCM) Institutional Animal Care and Use Committee (protocol number AN-4843) in compliance with the National Research Council Guide for the Care and Use of Laboratory Animals. Mice were bred and housed in micro-isolator cages with chow and water provided *ad libitum*, using a 12 hour light-dark cycle in the specific pathogen-free Transgenic Mouse facility. The experimental SJL mouse colonies were derived from a male SJL CCR2HT mouse (kind gift from Dr. William Karpus, Northwestern University Feinberg School of Medicine, Chicago, Illinois, U.S.A.)[14] mated with female SJL CCR2WT mice (purchased from The Jackson Laboratory, Bar Harbor, Maine, U.S.A.). Tail snip genomic DNA extracted using the Direct PCR lysis reagent was used to genotype mice by polymerase chain reaction (PCR) according to the manufacturer's instructions.

The following primer sequences detected the normal and neomycin resistance cassette-disrupted CCR2 alleles: CCR2: Sense GGTCATGATCCCTATGTGG, Anti-sense CTGGGCACCTGATTTAAAGG;

Neomycin cassette: Sense ATTGAACAAGATGGATTGCAC, Anti-sense CGTCCAGATCATCCTGATCGA [15]. Littermate CCR2HT breeding pairs produced first generation CCR2KO mice. CCR2KO, CCR2KO and CCR2WT, and CCR2WT mating pairs were used to generate experimental mice. CCR2 gene disruption was further verified by semi-quantitative reverse transcription PCR of splenocyte messenger RNA, with glyceraldehyde-3 phosphate dehydrogenase (GAPDH) serving as an internal control. The following primers were used: CCR2: Sense GGTCATGATCCCTATGTGG, Anti-sense CTGGGCACCTGATTTAAAGG; GAPDH: Sense CCCCCACATAGGGATCATGA, Anti-sense GATGCAGGGATGATGTTCTG [9], [15]. Digital images of ethidium bromide-stained agarose gels were generated using an AlphaImager HP image documentation system (Cell Biosciences, Santa Clara, California, U.S.A.) attached to a Sony ICX267AL 1.39 Megapixel CCD camera and processed using the AlphaView software (version 3.2.2.0) and Adobe Photoshop CS2 (Adobe Systems, San Jose, California, U.S.A.) software programs.

### Experimental autoimmune neuritis

8–12 week old female SJL CCR2WT, CCR2HT and CCR2KO littermates were used for these series of experiments. Sm-EAN was induced using subcutaneous injections of purified BPNM emulsified in CFA, (containing 1 mg/mL heat-inactivated *Mycobacterium tuberculosis* strain H37RA); as previously published [9], [10], [13]. Each mouse received a total of 2.5 mg of emulsified BPNM on its back in four locations under ketamine 100 mg/kg + xylazine 10 mg/kg anesthesia on the day of induction (day 0). Intraperitoneal injections of 200 ng pertussis toxin were administered on days 0 and 2 post-induction, with 100 ng recombinant mouse interleukin-12 administered on days 1, 2 and 3 post-induction. Daily weights and neuromuscular severity scores (NMSS; based on a published 6-point scale: 0 indicates normal strength, 1 tail paresis only, 2 mild-to-moderate fore or hind limb paresis, 3 severe fore or hind limb paresis, 4 mild-to-moderate fore and hind limb paresis and 5 severe fore and hind limb paresis) [9] were obtained from each mouse during the disease induction and effector phases, up until day 30 post-induction. Mice were euthanized either at disease onset (following demonstrable tail weakness; days 7–9 post-induction) or at expected maximal severity (days 28–30 post-induction) to harvest tissue for further analyses. 11 CCR2WT, 15 CCR2HT and 12 CCR2KO mice were studied in three independent experiments over a 6-month period.

In another series of experiments to determine the functional effect of CCR2 signaling blockade during the early effector phases of the disorder, 5 mg/kg CCR2 antagonist RS 102895 (Sigma Aldrich) dissolved in 20% hydroxypropyl-β-cyclodextrin (Tokyo Chemical Industry, Tokyo, Japan) was administered 4 times a day (total daily dose of 20 mg/kg) via i.p. injection [16] to female sm-EAN-affected CCR2 WT mice from days 13 to 17 post-induction for a total of 5 days. Apart from establishing functional relevance of CCR2 signaling following clinically apparent disease, these series of studies were designed to mimic a therapeutic drug trial. 20% hydroxypropyl-β-cyclodextrin was administered i.p. four times a day as negative treatment [vehicle] control while 400 mg/kg human IVIg (Carimune nanofiltered, CSL Behring, King of Prussia, Pennsylvania, U.S.A.), the current gold standard treatment for GBS, was administered i.p. once daily as therapeutic treatment control. This was performed to determine the efficacy of specific CCR2 drug inhibition relative to human IVIg in this model. Intracardiac puncture was performed following exposure of the chest cavity under deep anesthesia to obtain blood for automated complete blood counts with differential quantitation of leukocyte subsets prior to euthanasia. This was performed to determine the effect of CCR2 inhibitor RS 102895 on bone marrow function in sm-EAN. The BCM Center for Comparative Medicine performed the automated leukocyte counts. Mice were euthanized at expected maximal severity (days 28–30 post-induction) to harvest tissue for further analyses. Twenty-seven female SJL mice with behavioral evidence of sm-EAN (mild-to-moderate fore or hind limb weakness) were studied in two independent experiments over a 10-week period.

### Motor nerve electrophysiology

Bilateral dorsal caudal tail nerve (DCTN) and sciatic nerve (ScN) motor electrophysiology studies were performed on all mice at expected maximal severity under the plane of ketamine 100 mg/kg + xylazine 10 mg/kg anesthesia. Surface body temperatures of sedated mice were maintained >34°C using an external heating device. A portable Keypoint v5.11 electrodiagnostic system (Alpine Biomed Corporation, Fountain Valley, California, U.S.A.) with waveforms displayed on a Tecra S3 LCD monitor (Toshiba America, Irvine, California, U.S.A.) was used, as previously published [9], [17], [18]. Distal and proximal compound motor action potential (CMAP) amplitudes [in mV], conduction velocity [in m/s] and distal CMAP total waveform duration [in ms; measured from the initial deflection of the waveform from the baseline to the point at which the waveform returns back to baseline] were obtained for comparative analyses of axonal integrity and myelination between groups of experimental mice [9], [17], [18]. In general, CMAP amplitudes serve as a measure of axonal integrity, while conduction velocities and total waveform durations serve as measures of axon myelination, with conduction velocities reflective of large myelinated axonal transmission.

### Sciatic nerve morphometric analysis

Sciatic nerves were harvested from at least 6 mice per experimental group and immediately fixed in 3% buffered glutaraldehyde in 0.1 M phosphate buffer overnight and stored in 0.1 M phosphate buffer at room temperature until further processed. Nerves were post-fixed in 1% osmium tetroxide for 2 hours and embedded in epoxy resin. 1 μm semi-thin plastic embedded sections were stained with 1% toluidine blue in distilled water and mounted with glass coverslips for light microscopy as previously published [9], [18]. Images were collected with a Zeiss Axioskop Epifluorescent microscope equipped with an Axiocam MRc 5 digital camera. Quantitative analyses of total endoneurial area, total demyelinated area and % demyelinated area (% of demyelinated area relative to total endoneurial area) were performed by outlining the entire axial section of the sciatic nerve and areas containing axons with absent or reduced myelination on digital photomicrographs of at least 5 sections separated 50 μm apart per experimental mouse, using a micrometer-calibrated Zeiss Axiovision software program. Qualitative assessment of leukocyte infiltration, demyelination and axonal loss at expected maximal sm-EAN severity was also performed by a trained neuromuscular pathologist.

### Indirect immunohistochemistry

Indirect fluorescent immunohistochemistry was performed on serial 10 μm frozen acetone-fixed, sciatic nerve axial sections from at least 6 mice per experimental group at expected maximal severity, using previously published protocols [9], [18]. At least 4 sections separated by 30–50 μm were analyzed per experimental mouse. All primary antibodies were used at 1∶50 dilution, with secondary antibodies at 1∶500 dilution, unless otherwise stated. The total numbers of inflammatory mononuclear cells, numbers of monocytes/macrophages, T- and B-cells and their relative percentages per section were determined using the NIH Image J software program. To demonstrate TLR2 and TLR4 expression in sciatic nerves at disease onset, sequential immunofluorescent labeling was performed on the same slide in the dark. TLR2 and TLR4 were independently labeled along with galactocerebroside (GCB: Schwann cell/myelin marker, 5 μg/mL) adapting previously published protocols [13], [19]. Healthy female SJL CCR2WT mice were used as negative sm-EAN controls. Images were collected with a Zeiss Axioskop Epifluorescent microscope equipped with an Axiocam MRc 5 digital camera. Images were taken using the same exposure time settings for each fluorochrome. Images were initially processed using AlphaView software (version 3.2.2.0) and then cropped and merged using Adobe Photoshop CS2. Table 1 lists the primary and secondary antibodies used in these experiments.

**Table 1:** Antibodies used for immunohistochemistry and western blot.

Antigen	Antibody Isotype	Clone	Commercial Source
F4/80	Rat IgG2b	CI:A3-1	AbD Serotec
CD3	Rat IgG2b	C363.29B	SouthernBiotech
CD19	Rat IgG2a	6D5	SouthernBiotech
S100β	Rabbit polyclonal IgG	H-56	Santa Cruz
Neurofilament-H	Rabbit polyclonal IgG	H-100	Santa Cruz
TLR2	Rabbit polyclonal IgG	H-175	Santa Cruz
TLR4	Rabbit polyclonal IgG	M-300	Santa Cruz
Galactocerebroside	Mouse IgG3	mGalC	Millipore
CCL2	Goat polyclonal IgG	M-18	Santa Cruz
β-actin	Mouse IgG1	ACTBD11B7	Santa Cruz
Rat IgG	Goat IgG (H+L) FITC/TXRD	N/A	SouthernBiotech
Rabbit IgG	Goat IgG (H+L) FITC/TXRD	N/A	SouthernBiotech
Mouse IgG	Goat IgG (H+L) TXRD	N/A	SouthernBiotech
Rabbit IgG	Goat AffiniPure IgG (H+L) HRP	N/A	Jackson ImmunoResearch
Goat IgG	Donkey IgG (H+L) HRP	N/A	Santa Cruz
Mouse IgG	Goat IgG (H+L) HRP	N/A	Jackson ImmunoResearch

Abbreviations: FITC: fluorescein, H+L: heavy and light chain, HRP: horseradish peroxidase, N/A: not applicable, TXRD: Texas Red.

### Splenocyte proliferation assay

Splenocytes were immediately harvested from the spleens of healthy CCR2WT, CCR2HT and CCR2KO mice by mechanical dissociation and density centrifugation [20], with viability >95% by the trypan blue exclusion test. Nine mice per genotype were studied. 500,000 viable splenocytes from each mouse were cultured in 96-well Corning CellBIND plates using 100 μL of specialized medium (10% fetal bovine serum in RPMI-1640 with 1× penicillin-streptomycin, 2 mM L-glutamine, 1× non-essential amino acids and 25 mM HEPES) containing 100 ng BPNM, 100 ng phytohemagglutinin (PHA) or without mitogens for 4 days in a humidified incubator maintained at 37°C containing 95% air+ 5% CO_2_. 10–5000 ng of BPNM and PHA were used in separate assays prior to determining the most effective doses above. The 4-hour non-radioactive WST-1 proliferation assay was performed to determine the effect of BPNM on splenocyte proliferation *in vitro*. The optical density at 485 nm minus optical density at 595 nm is directly proportional to the number of viable cells [21], [22]. This series of experiments was designed to determine whether CCR2 gene disruption affects immune cell proliferation in response to BPNM *in vitro*.

### Splenocyte cytokine expression assay

15 million splenocytes from healthy CCR2WT, CCR2HT and CCR2KO mice were cultured in 6-well Corning CellBIND plates containing 1.5 mL of specialized medium with or without 3 μg of BPNM for 4 days in a humidified incubator maintained at 37°C containing 95% air+ 5% CO_2_. A total of 18 mice (6 per genotype) were studied. Supernatants were collected and stored at −80°C prior to analysis. This assay was performed to determine the effect of CCR2 gene disruption on systemic immune cell pro-inflammatory and anti-inflammatory cytokine secretion in response to BPNM *in vitro*. Splenocytes were also obtained from 3 CCR2WT, 3 CCR2HT and 3 CCR2KO mice 7 days following sm-EAN induction using BPNM. Total cytoplasmic and membrane proteins were isolated and stored at −80°C [23]–[25]. This assay was performed to determine the effect of CCR2 gene disruption on systemic immune cell intracellular pro-inflammatory and anti-inflammatory cytokine expression at the onset of sm-EAN *in vivo*. TNF-α, IFN-γ, IL-1β, IL-4, IL-6 and IL-10 levels were measured in equivalent supernatant or protein homogenate aliquots using the commercially available Millipore mouse cytokine multiplex assays in duplicate or triplicate. These assays were performed by the BCM Proteomics Core facility.

### Western blot

Snap frozen experimental mouse sciatic nerve specimens were homogenized using a disposal pestle device on ice [26], and total cytoplasmic and membrane proteins extracted using previously published protocols. Equal amounts of protein were denatured, reduced and separated by sodium dodecyl sulfate-polyacrylamide gel electrophoresis using the Bio-Rad MiniProtean III Apparatus, then electrotransfered to polyvinylidene fluoride membranes for western blot. Primary antibodies were used at a concentration of 1∶200, with secondary antibodies at 1∶10,000–20,000. Membranes were treated with Pierce Enhanced Chemiluminescence western blotting substrate plus detection reagents (Thermo Fisher Scientific, Rockford, Illinois, U.S.A.) and visualized by generating autoradiographs following film exposure from 1 minute to 1 hour using an SRX-101A film processor (Konica Minolta, Tokyo, Japan). TLR2, TLR4 and CCL2 expression were compared between CCR2 WT, CCR2HT and CCR2KO mice by semi-quantitative spot densitometric analyses of digital autoradiographs relative to β-actin expression, using previously described methods [23]–[25]. These experiments sought to determine whether CCR2 gene disruption had an effect on the peripheral nerve innate immune responses at the onset of sm-EAN, an effect on endogenous CCL2 secretion at disease onset and expected peak severity or both. Images were taken using an AlphaImager HP image documentation system (Cell Biosciences) attached to a Sony ICX267AL 1.39 Megapixel CCD camera, and were initially processed with the Zeiss Axiovision software and merged using Adobe Photoshop CS2. Table 1 lists the primary and secondary antibodies used in these experiments.

### Statistical analyses

The following statistical programs were used for data analyses: OpenStat, R version 2.13.1 (R Foundation, Vienna, Austria), Microsoft Office Excel 2003 and JMP version 8 (SAS Institute, Cary, North Carolina, U.S.A.). Mann-Whitney U-test or the Wilcoxon-Kruskall's Rank Sum Test was used to determine statistically significant differences between non-parametric variables while one- or two-tailed unpaired Student's/Welch's t-test (or analysis of variance for multiple comparisons) was used for parametric variables based on the Shapiro-Wilk test of normality (including measures of skew and kurtosis). Investigator-blinded analyses were performed for all parameters evaluated. Means are displayed, with variations of the mean depicted as standard errors. Statistical significance is defined as a p-value <0.05.

## Results

### Verification of CCR2 genotype in experimental mice

PCR of purified tail snip genomic DNA and splenocyte cDNA from breeding and experimental SJL mice verified CCR2 genotypes (Figure 1). CCR2KO and CCR2HT mice demonstrated similar viability at birth, reproductive capacity and lifespans compared to CCR2WT mice.

**Figure 1:** PCR verification of CCR2 genotype. Representative digital images of ethidium bromide-stained agarose gels of resolved tail snip genomic DNA (A and B) and splenocyte cDNA (C and D) demonstrate mouse CCR2 genotype. Mice that lack CCR2 genomic DNA (A) and express the neomycin cassette (B) are knockout (KO), while wild type (WT) mice express CCR2 without the neomycin cassette. Heterozygote (HT) mice express both. KO mouse splenocytes do not express CCR2 cDNA, in contrast to HT and WT mice (C). GAPDH serves as an internal loading control and housekeeping gene for splenocyte cDNA loading (D).

### CCR2 gene deletion significantly modulates sm-EAN incidence, onset and severity

Behavioral evidence of sm-EAN was observed in 8.3% of CCR2KO mice (1/12) compared to 100% of CCR2WT (11/11) and CCR2 HT (15/15) mice, with a disease onset of 20 days post induction observed in a single CCR2KO mouse compared to an average onset of 8.4 days with CCR2WT and 9.1 days with CCR2HT mice. There was no statistically significant difference in disease onset between CCR2HT and CCR2HT mice. Disease severity was significantly attenuated in CCR2KO mice. There is no appreciable difference observed between CCR2WT and CCR2HT mice, suggesting that CCR2KO mice are resistant to sm-EAN during the expected induction and effector phases of the disease (Figure 2A). CCR2KO mice demonstrated significantly faster DCTN and ScN motor conduction velocities and shorter total distal CMAP waveform durations than CCR2WT and CCR2HT mice, indicative of relative resistance to demyelination in both nerves. CCR2KO mice also demonstrated significantly larger DCTN distal CMAP amplitudes compared to CCR2 WT and CCR2HT mice. However, there was no significant difference observed in ScN distal CMAP amplitudes, suggesting reduced axonal injury in the DCTN only (Figures 2B–G). These data support the notion that CCR2KO mice may not develop a primary demyelinating neuropathy or may develop a very mild form of a demyelinating polyneuropathy with some axonal loss in some nerves compared to CCR2WT and CCR2HT mice. These series of experiments demonstrate the resistance of CCR2KO mice to sm-EAN suggesting a pathogenic role for CCR2 in acute peripheral nerve inflammatory demyelination. Representative electrophysiological waveforms demonstrating essential differences between the CCR2 genotypes at expected sm-EAN peak severity are shown in Figure 3.

**Figure 2:** Effect of CCR2 gene deletion on the behavioral features of sm-EAN. CCR2 gene deletion (CCR2KO) results in significantly delayed disease onset and markedly attenuated disease severity based on neuromuscular severity scores (NMSS), with no difference in disease onset or severity between CCR2WT and CCR2HT mice (A). Bar histographs of mean motor electrophysiology data from the bilateral dorsal caudal tail (DCTN; B–D) and sciatic (ScN; E–G) nerves obtained from each mouse at expected maximal severity support CCR2KO resistance to immune-mediated demyelination. Higher conduction velocities (a measure of large myelinated axon integrity; C and F) and shorter waveform durations (a measure of axonal conduction synchrony; D and G) are seen in CCR2KO compared to CCR2WT and CCR2HT mice. No significant differences are seen between the latter two genotypes for these parameters. CCR2KO mice demonstrate significantly higher DCTN compound motor action potential (CMAP) amplitudes (B), implying resistance to secondary axonal degeneration or distal conduction block in these nerves, without significant differences seen in the ScN (A). Four nerves were studied in each mouse. N = 38. * indicates p<0.05, N.S. not significant.

**Figure 3:** Effect of CCR2 gene deletion on the electrophysiologic features of sm-EAN. Digital motor nerve conduction waveforms from a CCR2WT and a CCR2HT mouse with severe sm-EAN and a CCR2KO mouse resistant to sm-EAN on day 30 post-induction are shown for the DCTN (A–C) and ScN (D–F). The upper waveforms (in green) are obtained after distal nerve stimulation, while the lower waveforms (in red) are obtained following proximal nerve stimulation. Numbers on the right above each waveform indicate stimulus current (in mA) utilized to achieve supramaximal nerve stimulation. Reduced amplitudes, slower conduction velocities and increased total waveform durations or waveform dispersion (a marker of axonal conduction dyssynchrony due to demyelination; black arrows) are more commonly seen in CCR2WT and CCR2HT mice compared to CCR2KO mice. Sensitivity  =  10 mV/division for the DCTN and 20 mV/division for the ScN, and sweep speed 2 ms/division for both studies. D = division.

Furthermore, indirect immunohistochemistry demonstrated reduced S100β staining (indicative of Schwann cell loss or demyelination) associated with F4/80+ monocyte/macrophage, CD3+ T-cell and CD19+ B-cell infiltration into sciatic nerves of sm-EAN-affected CCR2WT and CCR2HT mice compared to CCR2KO mice at expected peak severity (Figures 4A-O). Statistically significantly higher mean numbers of infiltrating cells were seen in CCR2WT and CCR2HT mice compared to CCR2KO mice. In addition, significantly higher mean infiltrating cell numbers were observed in CCR2WT compared to CCR2HT mice. Significant reductions in the mean counts and relative percentages of F4/80+ macrophages, CD3+ T-cells and CD19+ B-cells were observed in CCR2KO mice compared to CCR2WT and CCR2HT mice. Interestingly, significantly higher mean counts and percentage of F4/80+ macrophages were observed in CCR2WT mice compared to CCR2HT mice despite the observation that there was no difference in disease severity between these groups. No significant differences were seen in the mean counts and relative percentage of CD3+ T-cells and CD19+ B-cells between these mice (Figures 4P-X). These data suggest that complete CCR2 gene disruption attenuates inflammatory cell infiltration into peripheral nerves with resultant resistance to demyelination expected in sm-EAN. Partial CCR2 gene deletion significantly modulates F4/80+ monocyte/macrophage infiltration into the peripheral nerves without altering T-cell and B-cell infiltration. A threshold level of CCR2 gene transcription or messenger RNA translation may be necessary to facilitate sufficient effector monocyte infiltration into peripheral nerves to induce inflammatory demyelination during sm-EAN.

**Figure 4:** Effect of CCR2 gene deletion on the histopathological features of sm-EAN. Representative digital indirect fluorescent immunohistochemistry photomicrographs of 10 μm frozen acetone fixed, axial sciatic nerve sections show foci of demyelination (white asterisk) associated with mononuclear cell infiltrates in CCR2WT (A) and CCR2HT (F) mice, compared to the normal uniform honeycomb appearance seen with S100β staining (Schwann cell and myelin marker) [9] observed with CCR2KO mice (K). No obvious qualitative difference in axonal density (heavy chain neurofilament [NF-H] staining) is seen between the genotypes in these sections (B, G and L). Diffuse infiltration of F4/80+ monocytes/macrophages is seen in CCR2WT (C) and CCR2HT (H) mice, compared to a few foci observed in CCR2KO mice (M). Multiple foci of CD3+ T-cells and CD19+ B-cells are seen in CCR2WT (D and E) and CCR2HT (I and J) mice [white arrows], while these cells are rarely seen in CCR2KO mice (N and O). Cells are detected by the 4', 6-diamidino-2-phenylindole (DAPI) nuclear stain in all images. Scale bar  =  100 μm. Quantitative analyses show significant differences in the mean total number of mononuclear cells (DAPI+) between CCR2WT, CCR2HT and CCR2KO mice (P, S and V), with a significant step-wise reduction in mean numbers (Q) and percentages (R) of F4/80+ monocytes/macrophages with CCR2 gene allele deletion per section. Significant reduction in CD3+ T cell numbers (T) and percentages (U), as well as CD19+ B cell numbers (W) and percentages (X) per section is seen in CCR2KO relative to both CCR2WT and CCR2HT mice, with no significant differences between the latter two genotypes. At least 4 sections per mouse separated by > 30 μm were analyzed from 5 mice per genotype for each immune cell marker. * indicates p<0.05, N.S. not significant.

Qualitative assessment of semi-thin plastic embedded sciatic nerve sections demonstrated axonal demyelination associated with mononuclear cell infiltration and intra-endoneurial edema in CCR2WT and CCR2HT mice. These features were uncommon in CCR2KO mice (Figures 5A–C). Statistically significant increases in mean total endoneurial area, total demyelinated area and % demyelinated area relative to total endoneurial area were observed in CCR2WT and CCR2HT mice compared to CCR2KO mice. No significant differences were observed between CCR2WT and CCR2HT mice (Figures 5D–F). The increase in total endoneurial area observed in CCR2WT and CCR2HT mice is attributed to intra-endoneurial edema. These data show that CCR2KO resistance to sm-EAN was associated with reduced mononuclear leukocyte infiltration and inflammatory demyelination compared to CCR2WT and CCR2HT mice. Partial CCR2 deletion had no significant effect on the behavioral, electrophysiological and pathological features of sm-EAN. An important pathogenic role for CCR2 in sm-EAN is inferred, with a minimal threshold effect at or below the CCR2 gene translation or mRNA transcription in CCR2HT mice being necessary for uninhibited disease induction and manifestation. A question remains as to whether CCR2 has a direct pathogenic role in hematogenous leukocyte trafficking into peripheral nerves or acts indirectly by altering specific systemic and innate peripheral nerve immune responses to BPNM during the induction or effector phases in sm-EAN.

**Figure 5:** Effect of CCR2 gene deletion on sm-EAN associated inflammatory demyelination. Representative digital photomicrographs of toluidine-blue stained, 1 μm semi-thin axial plastic embedded mouse sciatic nerve sections show foci of demyelinated axons associated with infiltrated mononuclear cells (white asterisk) and intra-endoneurial edema (paler background; white arrow) in CCR2WT mice (A), with an example of more confluent demyelinated segments seen in a CCR2HT mouse (B). These are in contrast to the normal appearing honeycomb appearance of myelinated axons seen within the endoneurium of CCR2KO mice (C). Scale bar  =  100 μm. Quantitative analyses demonstrate statistically significant increase in mean total endoneurial area [associated with leukocyte infiltration and intra-endoneurial edema] (D), total demyelinated area (E) and percentage demyelinated area (F) per section in CCR2WT and CCR2HT mice compared to CCR2KO mice. No significant differences are seen between CCR2WT and CCR2HT mice. At least 30 sections separated by > 50 μm from 6 mice per genotype were analyzed. * indicates p<0.05, N.S. not significant.

### CCR2 gene deletion enhances relative BPNM-induced splenocyte proliferation *in vitro*

BPNM had little effect on mean total murine splenocyte proliferation *in vitro*, compared with PHA (Figure 6A–C). No significant differences were seen in the mean absolute splenocyte numbers 4 days after culture with and without BPNM (Figure 6D); however the mean proliferation index (the ratio of the number of splenocytes after culture with BPNM to basal culture conditions without BPNM for 4 days for each mouse) was statistically significantly higher in CCR2HT and CCR2KO mice compared to CCR2WT mice. No differences were seen between CCR2HT and CCR2KO mice (Figure 6E). These data suggest that partial or complete CCR2 gene disruption weakly enhanced relative murine splenocyte proliferation to BPNM *in vitro*. The similarities in splenocyte proliferation index between CCR2HT and CCR2KO mice imply that slight increases in splenocyte proliferation (as a possible protective effect) would not explain the observed resistance of CCR2KO to sm-EAN compared to CCR2HT and CCR2WT mice.

**Figure 6:** Effect of CCR2 gene deletion on BPNM-induced splenocyte proliferation *in vitro*. Bar histographs depicting the mean absorbance of cultured splenocytes (optical density at 485 nm minus optical density at 595 nm; directly proportional to the number of viable cells) following treatment with bovine peripheral nerve myelin (BPNM) or phytohemagglutinin (PHA) show no significant increases in mean absolute proliferation in response to BPNM irrespective of CCR2 genotype compared to basal culture conditions (A–D). Significantly increased splenocyte proliferation to PHA verifies splenocyte viability and proliferative capacity (A–C). Deletion of one or both CCR2 gene alleles is associated with a small but significant relative increase in mean BPNM-induced splenocyte proliferation relative to basal proliferation on a mouse-per-mouse basis *in vitro*, with no significant difference observed between CCR2HT and CCR2KO mice (E). N = 9 mice per genotype, with each assay performed in triplicate. * indicates p<0.05, N.S. not significant.

### CCR2 gene deletion does not significantly alter BPNM-induced splenocyte cytokine expression

Statistically significant differences were observed in the mean basal secreted TNF-α and IFN-γ levels by CCR2WT and CCR2HT mouse splenocytes compared with CCR2KO mice after 4 days of culture. There were no differences for these cytokines between CCR2WT and CCR2HT (Figures 7A and B). In addition, no significant differences were observed in basal IL-1β, IL-4 and IL-6 secretion between these CCR2 genotypes (Figures 7C–E). Significant mean differences were observed in basal IL-10 secretion between CCR2WT and both CCR2HT and CCR2KO, with no differences between CCR2HT and CCR2KO (Figure 6F). Importantly, BPNM did not significantly induce splenocyte cytokine secretion above basal levels after 4 days co-culture, with no significant differences seen between CCR2 genotypes (Figures 7G–L). Similarly, no significant differences were observed for the tested intracellular splenocyte cytokine levels at expected sm-EAN disease onset between CCR2WT, CCR2HT and CCR2KO mice (Figures 7M-R). Our data suggests that BPNM did not significantly induce specific pro-inflammatory or anti-inflammatory cytokine expression in splenocytes *in vitro* after 4 days in culture or *in vivo* at expected disease onset. The data interestingly imply that early alterations in systemic immune cell cytokine expression were less likely to be responsible for BPNM-induced sm-EAN. These data also suggest that the observed resistance of CCR2KO mice to sm-EAN was not due to attenuated pro-inflammatory or enhanced anti-inflammatory cytokine expression by systemic immune cells in response to BPNM at expected disease onset.

**Figure 7:** Effect of CCR2 gene deletion on BPNM-induced splenocyte cytokine expression *in vitro* and *in vivo*. Bar histographs representing mean levels of mouse splenocyte pro- and anti-inflammatory cytokine secretion under basal culture conditions and following treatment with BPNM *in vitro* (A–F) show statistically significantly reduced basal mean TNF-α (A) and IFN-γ (B) levels in CCR2KO compared to both CCR2WT and CCR2HT. Reduced basal mean IL-10 levels are seen in CCR2HT and CCR2KO mice compared to CCR2WT mice (F). There are no statistically significant differences in cytokine secretion following BPNM treatment for any of the tested cytokines in these CCR2 genotypes based on absolute numbers (A–F) or expression relative to basal levels on a mouse-per-mouse basis (activation index; G–L). Data from 6 mice per genotype were analyzed in duplicate. In addition, no statistically significant differences in intracellular splenocyte cytokine expression are seen between the CCR2 genotypes following *in vivo* sm-EAN induction with BPNM at expected disease onset (M-R). N = 3 mice per genotype, with assays performed triplicate. * indicates p<0.05; other comparisons are not significant and are not shown to maintain figure clarity.

### CCR2 gene deletion is not associated with changes in sciatic nerve TLR expression

TLR expression is indicative of innate immune activation in peripheral tissues [27]. TLR2 and TLR4 were expressed in the sciatic nerves of sm-EAN mice at expected disease onset, co-localizing with Schwann cells, based on GCB co-expression (Figure 8A–H). No significant differences in expression were observed between CCR2WT, CCR2HT and CCR2KO mice for both TLR2 (Figures 8I and J) and TLR4 (Figures 8K and L). CCR2KO mice demonstrated similar endogenous innate immune activation in peripheral nerves in response to BPNM to CCR2HT and CCR2WT mice at expected sm-EAN disease onset. These data suggest that high relative levels of endogenous peripheral nerve TLR2 and TLR4 expression were temporally associated with sm-EAN disease onset; however the observed resistance of CCR2KO mice to sm-EAN was not as a consequence of aberrant innate peripheral nerve immune activation in response to BPNM in peripheral nerves.

**Figure 8:** Effect of CCR2 gene deletion on Toll-like receptor (TLR) expression at expected sm-EAN onset. Representative merged digital indirect fluorescent immunohistochemistry photomicrographs of 10 μm frozen acetone fixed, axial sciatic nerve sections stained to detect galactocerebroside (GCB; Schwann cell and myelin marker; red) and TLR2 (A–D; green) or TLR4 (E–H; green) demonstrate increased TLR expression co-localizing with Schwann cells (white arrows: yellow/orange immunoreactivity) in all CCR2 genotypes at sm-EAN onset, prior to significant mononuclear cell infiltration, compared to control mice not affected with sm-EAN. TLR2 or TLR4 expression may be multifocal (B and G), focally diffuse (D and F) or honeycomb (C and H) in early sm-EAN. Representative digital autoradiographs following western blot of sciatic nerve protein homogenates demonstrate similar TLR2 (I) and TLR4 (K) expression for all CCR2 genotypes, using β-actin as an internal protein loading control. Molecular weights in KDa are in brackets. No statistically significant differences are seen in TLR2 or TLR4 expression between the CCR2 genotypes based on semi-quantitative spot densitometry analyses relative to β-actin (J and L). N = 3 mice per genotype, with assays performed in duplicate experiments. WT =  wild type, HT = heterozygote, KO = knockout; N.S. not significant

### Sciatic nerve CCL2 expression is not altered at expected disease onset by CCR2 gene deletion

CCL2, the major ligand for CCR2 [28], is expressed in the peripheral nerves of human GBS patients and sm-EAN affected mice [5], [13]. CCL2 expressed on the luminal membrane of endoneurial microvessels could facilitate CCR2+ hematogenous leukocyte infiltration into peripheral nerves. Alterations in CCL2 expression between CCR2 genotypes at disease onset could explain the observed differences between CCR2KO and CCR2WT and CCR2HT mice. However, no statistically significant differences were seen in total relative CCL2 expression in the sciatic nerves of CCR2WT, CCR2HT and CCR2KO mice at expected disease onset (Figures 9A and B). This implies that the observed reduction in hematogenous mononuclear cell infiltration (monocytes/macrophages>T-cells>B-cells) in CCR2KO mice following sm-EAN induction was not due to altered peripheral nerve CCL2 expression at disease onset. Interestingly, there was a small, but a statistically significant increase in mean relative sciatic nerve CCL2 expression observed in CCR2HT mice compared to both CCR2WT and CCR2KO at expected peak severity. No difference was observed in CCL2 expression between CCR2WT and CCR2KO mice (Figures 9C and D).

**Figure 9:** Effect of CCR2 gene deletion on CCL2 expression at expected sm-EAN onset and maximal severity. Representative digital autoradiographs following western blot of sciatic nerve protein homogenates demonstrate CCL2 expression as presumed dimers (d), tetramers (t) and higher-order oligomers (o) at expected disease onset in all CCR2 genotypes, with β-actin serving as an internal protein loading control (A). CCL2 oligomerization is expected during *in vivo* secretion, and this has been demonstrated by western blot [31]. No statistically significant differences are seen in mean total CCL2 expression at disease onset between the CCR2 genotypes based on semi-quantitative spot densitometry analyses relative to β-actin (B). At expected maximal severity, CCL2 expression predominantly occurs as presumed tetramers (t) and higher-order oligomers (o) with loss of dimer expression in all CCR2 genotypes (C). A small, but statistically significant increase in mean total CCL2 expression is observed in CCR2HT compared to both CCR2WT and CCR2KO, with no difference observed between CCR2WT and CCR2KO mice (D). Numbers in A and C represent molecular weights in kDa. Data are obtained from three mice per genotype, in quadruplicate for expected disease onset experiments and triplicate for expected maximal severity experiments. WT =  wild type, HT = heterozygote, KO = knockout; N.S. not significant.

Mean CCL2 expression may be slightly reduced in CCR2WT compared to CCR2HT due to higher receptor-mediated ligand internalization and degradation following CCL2-mediated signaling (as there was an increased number of infiltrated cells with expected higher receptor density per cell in CCR2WT mice compared to CCR2HT mice), while CCR2KO may have lower mean CCL2 levels than CCR2HT mice owing to reduced numbers of secreting infiltrated mononuclear cells as a consequence of reduced trafficking into peripheral nerves, despite unaffected Schwann cell secretion [28]–[31]. Since CCL2 is similarly expressed in the sciatic nerves at sm-EAN disease onset irrespective of genotype, CCR2 gene deletion with resultant abrogated F4/80+ monocyte transmigration across the blood-nerve barrier into peripheral nerves is the most likely explanation for the observed CCR2KO mouse resistance to sm-EAN. Altered monocyte infiltration in CCR2KO mice has been previously described following mouse sciatic nerve transection [32].

Adoptive transfer or parabiosis experiments following bone marrow ablation in experimental models [33] provide an avenue to determine the functional significance of specific mononuclear cell populations in the pathogenesis of immune-mediated disorders. Functional assays using specific small molecular antagonists also provide useful mechanistic information without altering the immune status or disease susceptibility of experimental mice. Furthermore, these function neutralizing experiments provide some insight to the effect of modulating potentially relevant signaling pathways in sm-EAN that could directly translate towards human treatment trials.

### Pharmacologic CCR2 blockade ameliorates sm-EAN in female SJL mice

Treatment of sm-EAN affected mice with a total of 20 mg/kg CCR2 antagonist RS 102895 for 5 consecutive days during the early effector stage significantly reduced disease severity to near normal within 48 hours after the first dose was administered. This treatment effect persisted for up to 2 weeks relative to vehicle controls. This drug was also significantly more efficacious than human IVIg administered via i.p. injection during the same time period. Significant differences in NMSS were also observed with human IVIg treatment relative to vehicle control 6 days after completing treatment (Figure 10A). CCR2 inhibition was associated with faster motor conduction velocities and shorter total distal CMAP waveform durations compared to vehicle treated and human IVIg treated control mice (suggesting reduced axonal demyelination), and significantly larger distal CMAP amplitudes compared to vehicle control treated mice only (suggesting reduced axonal injury or loss) at expected peak severity. Human IVIg treated mice had significantly faster motor conduction velocities and higher amplitudes than vehicle treated mice, without significant differences in total distal CMAP duration, suggesting reduced axonal injury or loss and residual or persistent large myelinated axonal demyelination relative to vehicle controls (Fig 9B–G). These data suggest that RS 102895 rapidly arrests peripheral nerve demyelination and axonal injury during the early effector phases of sm-EAN, while human IVIg demonstrates a delayed treatment effect with more significant protection against axonal injury than demyelination. These data support a functional role for CCR2-mediated signaling pathways in sm-EAN pathogenesis during the effector phase, as well as the treatment efficacy of 20 mg/kg RS 102895 in sm-EAN. Representative electrophysiological waveforms demonstrating the differences between CCR2 inhibitor treated and untreated mice, compared with human IVIg treated mice are shown in Figure 11.

**Figure 10:** Effect of CCR2 drug inhibition on the behavioral features of sm-EAN. Treatment with RS 102895, a specific CCR2 inhibitor (CCR2INB; N = 9) from days 13–17 post-induction (early effector phase) results in rapid and persistent improvement in muscle strength supported by significantly lower mean NMSS compared to Vehicle (N = 10) and human IVIg (N = 8) treated mice. Statistically significant differences are observed between Human IVIg and Vehicle-treated mice from day 23 post-induction (6 days after completing drug therapy) with no further worsening in human IVIg treated mice (A). The yellow bar indicates the drug treatment phase, * indicates p<0.05 relative to both Vehicle and IVIg treated mice, # indicates p<0.05 comparing human IVIg and Vehicle treated mice. Bar histographs summarizing mean motor electrophysiology from the bilateral dorsal caudal tail (DCTN; B–D) and sciatic (ScN; E–G) nerves obtained from each mouse at expected maximal severity demonstrate significantly higher conduction velocities and shorter total waveform durations following CCR2INB treatment compared to Vehicle and human IVIg (hIVIg) treated mice. CCR2INB and hIVIg treatment result in higher compound motor action potential (CMAP) amplitudes than Vehicle treated controls (implying protection from axonal degeneration or distal conduction block), with no significant differences seen between the former two treatments (B and E). Despite small but significantly increased mean conduction velocities following hIVIg treatment compared to Vehicle controls (C and F), no significant differences are observed in total waveform duration (D and G) implying residual axonal dyssynchrony (demyelination or early remyelination) following IVIg treatment. * indicates p<0.05, N.S. not significant

**Figure 11:** Effect of CCR2 drug inhibition on the electrophysiologic features of sm-EAN. Digital motor nerve conduction waveforms from Vehicle, CCR2 inhibitor RS 102895-treated, and human IVIg-treated mice with sm-EAN mice on day 30 post induction are shown for the DCTN (A–C) and ScN (D–F). The upper waveforms (in green) are obtained after distal nerve stimulation, while the lower waveforms (in red) are obtained following proximal nerve stimulation. Numbers on the right above each waveform indicate stimulus current (in mA) utilized to achieve supramaximal nerve stimulation. Reduced CMAP amplitudes (open white arrows), slower conduction velocities and waveform dispersion (evidence of axonal conduction dyssynchrony due to demyelination; black arrows) are more commonly seen in Vehicle and human IVIg-treated mice compared to RS 102895 treated mice. Sensitivity  =  10 mV/division for the DCTN and 20 mV/division for the ScN, with a sweep speed 2 ms/division for both studies. D = division.

Treatment with RS 102895 was not associated with statistically significant differences in mean total white cell count, mean absolute monocyte, lymphocyte and neutrophil counts, or mean monocyte, lymphocyte and neutrophil differential (%) counts compared to vehicle control and human IVIg treated mice with sm-EAN at expected maximal severity (Table 2). These data imply that RS 102895 does not induce significant bone marrow suppression or cause depletion of the major leukocyte subpopulations in sm-EAN affected mice, further supporting efficacy at the level of hematogenous leukocyte trafficking into peripheral nerves.

**Table 2:** Comparative mean complete blood counts and leukocyte subset differentials in treated sm-EAN mice.

Parameter	Vehicle	RS 108295	Human IVIg
**Total white cell count (per μL)**	3338 (±590)	2735 (±466)	3843 (±563)
**Absolute monocyte count (per μL)**	26 (±10)	20 (±7)	24 (±5)
**Monocyte differential count (%)**	0.92 (±0.46)	0.65 (±0.11)	0.74 (±0.16)
**Absolute lymphocyte count (per μL)**	2559 (±568)	1854 (±413)	2543 (±473)
**Lymphocyte differential count (%)**	73.48 (±2.79)	63.75 (±6.16)	63.80 (±4.00)
**Absolute neutrophil count (per μL)**	554 (±76)	608 (±96)	1054 (±209)∧
**Neutrophil differential count (%)**	19.80 (±2.79)	18.29 (±3.19)	27.60 (±4.19)

Numbers in brackets represent standard errors of the means. N = 10 for vehicle, 8 for CCR2 inhibitor RS 108295 and 7 for human IVIg treated mice. ∧ Indicates p-value <0.05 relative to vehicle controls.

Indirect immunohistochemistry demonstrated reduced S100β staining (indicative of Schwann cell loss or demyelination) and neurofilament-H staining (indicative of axonal loss) associated with reduced F4/80+ monocyte/macrophage and CD3+ T-cell infiltration in the sciatic nerves of RS 102895-treated sm-EAN mice compared to vehicle and IVIg treated controls at expected peak severity (Figs 12A-L). These data support the notion that the observed drug efficacy was secondary to reduced hematogenous CCR2+ mononuclear leukocyte infiltration into peripheral nerves, with protection against the expected progressive inflammatory demyelination and axonal injury. Qualitative assessment of 1 μm semi-thin plastic embedded sciatic nerve sections demonstrated near absence of mononuclear leukocyte infiltration, demyelination and axonal loss following CCR2 inhibition compared to vehicle and IVIg treated mice. Clusters of thinly myelinated regenerating axons were more commonly observed following human IVIg treatment compared to vehicle control (Fig 13A–F). These data further support the functional role of CCR2 signaling in sm-EAN pathogenesis during the effector phase, as well as the efficacy of small molecular CCR2 antagonism in sm-EAN. Our data suggests a potential therapeutic role of CCR2 antagonists in acute severe immune-mediated demyelinating inflammatory neuropathies such as AIDP.

**Figure 12:** Effect of CCR2 drug inhibition on the histopathological features of sm-EAN. Representative digital indirect fluorescent immunohistochemistry photomicrographs of 10 μm frozen acetone fixed, axial sciatic nerve sections show disorganized or reduced S100β staining intensity indicative of demyelination (double white asterisk) associated with or without mononuclear cell infiltrates in Vehicle (A) and human IVIg treated (I) mice compared to the uniformly intense honeycomb appearance observed in CCR2 inhibitor (CCR2 INB) treated mice (E). The thin honeycomb background appearance seen in several regions of human IVIg treated mouse sections may also reflect early remyelination. Qualitative analyses suggest a reduction in large and small myelinated axon density in vehicle controls, associated with foci of mononuclear cells in some instances (white asterisk; B) compared to CCR2INB (F) and human IVIg treated (J) mice based on heavy chain neurofilament [NF-H] staining. Focal infiltration of F4/80+ monocytes/macrophages (white arrows), the predominant leukocyte subpopulation in sm-EAN, is seen in Vehicle controls (C). Fewer foci are seen following CCR2INB (G) and IVIg (K) treatment. Similarly, scattered foci of CD3+ T cells (white arrows) seen in Vehicle-treated controls (D) become less prevalent following CCR2INB (H) and IVIg (L) treatment. Fewer infiltrated mononuclear cells are observed with CCR2INB treatment compared to IVIg treatment. Cells are detected by the DAPI nuclear stain in all images. Scale bar  =  100 μm.

**Figure 13:** Effect of CCR2 drug inhibition on sm-EAN-associated inflammatory demyelination. Representative digital photomicrographs of toluidine-blue stained, 1 μm semi-thin plastic embedded axial sections of mouse sciatic nerves show multiple foci of demyelinated axons associated with infiltrated mononuclear cells (double white asterisk) in vehicle controls (A), compared to the preserved myelin architecture and lack of inflammation seen in CCR2INB treated mice (B). Clusters of thinly myelinated axons (double black asterisk) surrounded by large myelinated axons, suggestive of recent multifocal axonal injury and repair are commonly seen in human IVIg-treated mice, associated with scattered foci of mononuclear cells (black arrows; C). Higher magnification digital photomicrographs further demonstrate the mononuclear cell-mediated demyelination in Vehicle-treated controls as expected in untreated sm-EAN (white arrows). Active leukocyte extravasation at an endoneurial microvessel (EMV) is also seen (D). Foci of mononuclear cells (white arrow) are rarely seen in CCR2INB treated (white arrow; E); these are more common in human IVIg treated mice (black arrows; F). Scale bar  =  100 μm (A–C), 50 μm (D–F).

## Discussion

This study demonstrates a functional role of CCR2 in sm-EAN immunopathogenesis, implying a potential pathogenic role for CCL2/CCR2 signaling in AIDP. The data support a direct role of CCR2 in pathogenic mononuclear cell trafficking into peripheral nerves during immune-mediated injury, similar to observations in other inflammatory disorders [28]. Partial CCR2 deletion did not affect disease onset and severity despite the reduced numbers of infiltrating monocytes/macrophages observed in the peripheral nerves of affected mice, suggesting that at least 50% of expected CCR2 gene transcription is pathologically sufficient in sm-EAN. Interestingly, activation of peripheral nerve innate immune responses was more evident than systemic (splenocyte) immune activation in response to BPNM at expected disease onset, suggesting an important direct role for Schwann cells in the initiation of restricted peripheral nerve immune-mediated injury in this model [5], [13], [27], [34], [35]. The efficacy of a systemically administered, specific CCR2 small molecular antagonist several days after disease onset provided further mechanistic evidence and proof-of-concept to support testing leukocyte trafficking inhibitors such as chemokine receptor antagonists as target-specific therapies in AIDP.

A previous study evaluating chemokine receptor CCR5 in murine P0 peptide 180-199-induced EAN (a less robust and reliable mouse model than sm-EAN) demonstrated lack of disease protective effect, based on clinical course or severity of EAN, levels of spleen mononuclear cell response, or profile of infiltrating macrophages and T-cells into the cauda equina [36]. The authors attributed the lack of effect to a compensatory increase in CCL4 and CXCL10 in knockout mice compared to the wild type controls. Another potential explanation is redundancy in CCR5-mediated signaling pathways *in vivo*, as CCL5 can also signal through CCR1 and CCR3. Therefore, that study does not completely exclude a role for CCL5 in EAN pathogenesis [3], [13], [37]. However, those observations could also support the notion that another chemokine signaling pathway, such as CCL2/CCR2 is more relevant to EAN disease pathogenesis. Our study demonstrates a sufficient pathogenic role for CCR2 in sm-EAN.

CXCL10/CXCR3 signaling has also been implicated in GBS pathogenesis based on a report that demonstrated elevated CSF CXCL10 levels in GBS patients compared to controls, with CXCL10 messenger RNA co-localized to peripheral nerve vascular endothelium using *in situ* hybridization techniques [38]. Since CXCL10 signals via a single chemokine receptor CXCR3 which expressed on CD4+ T-helper 1 cells [39], the study proposed a role for CXCL10 in recruiting helper T-cells from circulating blood into peripheral nerves in GBS. CXCL10 has been shown to co- localize with murine endoneurial microvessels, with infiltrated CXCR3+ T-cells demonstrated at maximal severity in sm-EAN [13]. Primary human endoneurial endothelial cells (that form the blood-nerve barrier) also secrete CXCL10 constitutively *in vitro*, with increased expression observed following physiological cytokine stimulus [24]. In addition, small subsets of circulating human (∼20–25%) and infiltrated mouse CD3+ T-cells in sm-EAN are also CCR2+ [11], [13]. Our study demonstrated fewer CD3+ T-cells in CCR2KO mice compared to CCR2WT and CCR2HT mice, with no difference between the latter two genotypes. This observation may suggest a pathogenic role for CCR2+ CXCR3+ CD3+ T-cells in sm-EAN or an important role for peripheral nerve infiltrated CCR2+ monocyte/macrophage-dependent recruitment of pathogenic CXCR3+ CD3+ T-cells in this model.

We recently demonstrated the importance of α_M_β_2_-integrin (CD11b)-intercellular adhesion molecule-1 signaling pathways in GBS patient-derived mononuclear leukocyte trafficking *in vitro* using a flow- dependent human blood-nerve barrier model [24]. Interestingly, >99% of circulating GBS patient-derived CD14+ monocytes were CD11b+, and monocytes were the most prevalent firmly adherent or migrated leukocyte subpopulation observed (consistent with *in situ* GBS peripheral nerve studies). TNF-α and IFN-γ-stimulated confluent primary endoneurial endothelial cells in culture (i.e. the *in vitro* human blood-nerve barrier) also expressed CCL2 *de novo* in the referenced study [24]. Taking into account that most circulating monocytes are CCR2+ and our data using gene knockouts and pharmacologic blockade in sm-EAN, we speculate that CCL2/CCR2 signaling could drive pathogenic CD14+ CD11b+ CCR2+ monocyte trafficking into the endoneurium at the blood-nerve barrier in AIDP. Further studies are needed to evaluate this hypothesis using the flow-dependent *in vitro* human blood- nerve barrier model, and decipher whether combined chemokine receptor, integrin inhibition or both could be more efficacious (or detrimental) in treating severe peripheral nerve inflammatory demyelination. In addition, the specific chemokines responsible for recruiting regulatory T-cells and anti-inflammatory monocytes during GBS recovery are unknown. Such knowledge could further guide therapeutic strategies to limit peripheral neuroinflammation and promote peripheral nerve recovery in GBS and related disorders.

AIDP, a predominantly monophasic disorder with potentially serious consequences, provides an excellent opportunity to evaluate chemokine receptor blockade efficacy against currently approved therapies such as IVIg in patients with acute peripheral neuroinflammation using well-defined short and long-term outcome measures. Although chemokine biology during inflammation can be complex [40], [41], representative animal models typically require aggressive induction protocols with features that differ from the human disease and challenges exist in translating therapeutic observations from EAN models towards successful therapies supported by human GBS clinical trials [7], this study, guided by human observational data, suggests a key functional role for CCR2 in acute demyelinating peripheral neuritis, and as a consequence, provides mechanistic data that furthers our understanding of pathogenic hematogenous mononuclear cell trafficking in sm-EAN and possibly AIDP.
